The article "Suppression of MMP-2 Attenuates TNF-α Induced NF-κB Activation and Leads to JNK Mediated Cell Death in Glioma" was retracted in 2025. Reasons: duplicated images; overlap with earlier publications; unreliable data; unreliable results or conclusions.

# Suppression of MMP-2 Attenuates TNF-α Induced NF-κB Activation and Leads to JNK Mediated Cell Death in Glioma

**DOI:** 10.1371/journal.pone.0019341

**Published:** 2011-05-04

**Authors:** Divya Kesanakurti, Chandramu Chetty, Praveen Bhoopathi, Sajani S. Lakka, Bharathi Gorantla, Andrew J. Tsung, Jasti S. Rao

**Affiliations:** 1 Departments of Cancer Biology and Pharmacology, University of Illinois College of Medicine at Peoria, Peoria, Illinois, United States of America; 2 Department of Neurosurgery, University of Illinois College of Medicine at Peoria, Peoria, Illinois, United States of America; The University of Kansas Medical Center, United States of America

## Abstract

**Background:**

Abrogation of apoptosis for prolonged cell survival is essential in cancer progression. In our previous studies, we showed the MMP-2 downregulation induced apoptosis in cancer cell lines. Here, we attempt to investigate the exact molecular mechanism of how MMP-2 depletion leads to apoptosis in glioma xenograft cell lines.

**Methodology/Principal Findings:**

MMP-2 transcriptional suppression by MMP-2siRNA (pM) induces apoptosis associated with PARP, caspase-8 and -3 cleavage in human glioma xenograft cells 4910 and 5310. Western blotting and cytokine array showed significant decrease in the cellular and secreted levels of TNF-α with concomitant reduction in TNFR1, TRADD, TRAF2, RIP, IKKβ and pIκBα expression levels resulting in inhibition of p65 phosphorylation and nuclear translocation in pM-treated cells when compared to mock and pSV controls. In addition MMP-2 suppression led to elevated Fas-L, Fas and FADD expression levels along with increased p38 and JNK phosphorylation. The JNK-activity assay showed prolonged JNK activation in pM-transfected cells. Specific inhibition of p38 with SB203580 did not show any effect whereas inhibition of JNK phosphorylation with SP600125 notably reversed pM-induced cleavage of PARP, caspase-8 and -3, demonstrating a significant role of JNK in pM-induced cell death. Supplementation of rhMMP-2 counteracted the effect of pM by remarkably elevating TNF-α, TRADD, IKKβ and pIκBα expression and decreasing FADD, Fas-L, and phospho-JNK levels. The EMSA analysis indicated significant reversal of pM-inhibited NF-κB activity by rhMMP-2 treatment which rescued cells from pM-induced cell death. *In vivo* studies indicated that pM treatment diminished intracranial tumor growth and the immuno histochemical analysis showed decreased phospho-p65 and enhanced phospho-JNK levels that correlated with increased TUNEL-positive apoptotic cells in pM-treated tumor sections.

**Conclusion/Significance:**

In summary, our study implies a role of MMP-2 in the regulation of TNF-α mediated constitutive NF-κB activation and Fas-mediated JNK mediated apoptosis in glioma xenograft cells *in vitro* and *in vivo*.

The article "Suppression of MMP-2 Attenuates TNF-α Induced NF-κB Activation and Leads to JNK Mediated Cell Death in Glioma" was retracted in 2025. Reasons: duplicated images; overlap with earlier publications; unreliable data; unreliable results or conclusions.

## Introduction

Despite recent advances in treatment strategies, glioblastomas (GBM) are the most aggressive and deadliest form of primary brain tumors. These tumors remain incurable, and patients have a mean survival of 12 months after diagnosis [1]. Many factors support the highly treatment-resistant and persistent nature of GBM. Genetic abnormalities can defend the tumor from conventional therapies, the blood-brain barrier limits the entry of chemotherapeutic agents to tumors, and GBM have highly invasive potential with increased extracellular matrix (ECM) disruption [2]–[4]. The ECM disruption is achieved in part by the action of a group of serine-, cysteine- and metallo-proteases, among which matrix metalloproteases (MMPs), are zinc-dependent endopeptidases involved in the inclination of tumor cells to overrun normal tissues and to metastasize to distant sites [5], [6]. Among MMP family members, MMP-2 contains fibronectin domains for collagen binding and preferentially degrades basement membrane components such as type-IV collagen, which ultimately regulate cell migration and proliferation during tumor invasion [6]. The expression and activities of MMPs are increased in almost all human malignancies and are associated with advanced metastatic tumor stage and poor survival [7].

RNA interference (RNAi) is accomplished by different classes of small RNAs including microRNAs (miRNAs), small interfering RNAs (siRNAs) and Piwi-interacting RNAs (piRNAs) [8]. Among these, siRNAs which are short stretches of double-stranded RNA molecules are employed in specific knockdown of desired genes thus being widely used to investigate gene function with a future potential as therapeutic agents in the treatment of various diseases such as cancers [9]. Here, we attempted to evaluate the effect of targeted silencing of the MMP-2 gene using siRNA, and molecular mechanism in relation to apoptotic cell death of glioma both *in vitro* and *in vivo*.

The pro-inflammatory cytokine tumor necrosis factor-α (TNF-α) regulates various signaling pathways in proliferation, apoptosis, and inflammation through the activation of phospholipases, mitogen-activated protein kinases and NF-κB [10], [11]. The pleotropic biological functions of TNF-α are mediated through its cognate receptors TNFR1 and TNFR2, which activate various signalling pathways predominantly through TNFR1 [12]. The adaptor protein TRADD recruits additional adaptor proteins such as TRAF2, FADD and RIP [10], [13]. The TNF-α mediated functions emanate from TRADD, which transduces signals to different effectors such as IκB kinase (IKK), Janus N-terminal Kinase (JNK) and caspases [10]. The distinct role of TRADD in proliferation and apoptosis through binding with TRAF2 and FADD has been previously elucidated. TRADD directly interacts with TRAF2 at its N-terminal region, and this interaction is essential for cell survival through NF-κB signaling and efficient inhibition of apoptosis [12]. Activation of NF-κB through inhibitory phosphorylation of IκB by IKK complex leads to the nuclear translocation of NF-κB, where it stimulates the transcription of target genes that are involved in immune responses, inflammation and cell survival [14], [15]. It has been demonstrated that NF-κB controls the expression of various anti-apoptotic proteins including XIAP, IAP and gadd45α which inhibit caspase-dependent apoptosis and also encode target genes that inhibit c-Jun N-terminal kinase (JNK) activation [16]–[19]. On the other hand, Fas (APO-1/CD95) is a cell surface death receptor and upon Fas-ligand binding and activation, the procaspase-8 is recruited onto the Fas complex through FADD [20]. Cleavage and activation of pro caspase-8 induces activation of effector caspases-3 and -7 as well as Bid, which initiates the apoptotic machinery. The receptor interacting protein (RIP) is a kinase recruited to TNFR1-TRADD complex essential for activation of NF-κB signalling and the downregulation and cleavage of RIP from TNFR1 complex leads to inhibition in NF-κB activation and induces apoptosis [21]–[23].

The article "Suppression of MMP-2 Attenuates TNF-α Induced NF-κB Activation and Leads to JNK Mediated Cell Death in Glioma" was retracted in 2025. Reasons: duplicated images; overlap with earlier publications; unreliable data; unreliable results or conclusions.

The mitogen activated protein kinase (MAPK) family has three components: extracellular signal regulated kinase cascade, JNK cascade and p38 MAPK cascade. The c-Jun N-terminal kinase (JNK) is a serine/threonine protein kinase activated by a variety of extracellular stimuli such as UV and ionizing radiation, heat shock, inflammatory cytokines, metabolic inhibitors and osmotic or redox shock leading to cell death [24]. JNK is involved in several forms of cell-specific and stress-induced apoptosis, which are dependent on cell type and stimulus. It phosphorylates serine 63 and 73 at the N-terminal domain of c-Jun, thus activating the transcriptional activity of AP-1 [25]. The inhibition of NF-κB activation is required for prolonged JNK activation, which simultaneously results in apoptosis [16], [25], [26]. Several studies showed the role of JNK activation in the accomplishment of Fas signaling induced cell death [27]–[29].

Our previous studies with MMP-2 downregulation activated TIMP-3 induced Fas/CD95 mediated extrinsic apoptotic pathway and enhanced radiosensitivity in lung adenocarcinoma cells [30]–[32]. Our studies also indicated the siRNA mediated MMP-2 downregulation led to apoptosis in human glioma xenograft cells [32]. In the current study, we provide further insights in to the molecular mechanism underlying siRNA mediated MMP-2 depletion-induced apoptosis in human glioma xenograft cells 4910 and 5310 both *in vitro* and *in vivo*. We observed that the transcriptional suppression of MMP-2 inhibited TNF-α induced IKKβ/pIκBα mediated NF-κB activation by decreasing TRADD-TRAF2 interactions in xenograft cell lines. Here, we report concomitant activation MAP kinases, JNK and p38 and a role of JNK activation but not p38 in MMP-2siRNA induced apoptosis.

The article "Suppression of MMP-2 Attenuates TNF-α Induced NF-κB Activation and Leads to JNK Mediated Cell Death in Glioma" was retracted in 2025. Reasons: duplicated images; overlap with earlier publications; unreliable data; unreliable results or conclusions.

## Results

### MMP-2siRNA (pM) downregulates MMP-2 expression and activity in 4910 and 5310 cells

We transfected 4910 and 5310 cells with CMV promoter-driven MMP-2siRNA in pcDNA3.0 (pM) and determined the levels of MMP-2 using gelatin zymography, Western blotting, RT-PCR and immunofluorescence analyses. Conditioned media from pM-treated cells showed reduced gelatinase activity in comparison to mock and pSV-treated 4910 and 5310 cells (69.1±2.5% and 68.6±2.4%, respectively) (Fig. 1A). We observed substantial decrease in the MMP-2 expression up to 70.2±2.6% and 69.4±3.3% in pM-treated 4910 and 5310 cells as compared to mock and pSV treatments by Western blotting (Fig. 1B). Transcriptional levels of MMP-2, as assessed by RT-PCR, confirmed the decreased expression levels of MMP-2 up to 68.2±3.0% in pM-transfected 4910 cells and 69.0±2.2% in pM-transfected 5910 cells as compared to mock and pSV-treated counterparts (Fig. 1C). Quantification of relative expression level and gelatinolytic activity of MMP-2 showed significant decrease upon pM treatment at *p*<0.01. Immunofluorescence studies showed high expression levels of MMP-2 in mock- and pSV- treated 4910 and 5310 cells (Fig. 1D). The quantification of relative fluorescence intensity indicated a significant decrease in the MMP-2 expression upon pM treatment at 72 h (*p*<0.01).

**Figure 1:** Effect of RNA interference on MMP-2 expression in human xenograft cell lines 4910 and 5310. Different treatments included control (mock), pSV (scrambled vector), pM (pMMP-2Si, pcDNA3.1 vector containing siRNA sequence for MMP-2). A. Gelatin zymography of extracellularly secreted MMP-2 in to tumor conditioned medium at 72 h post-transfection. The bar diagrams below represent the quantification of gelatinolytic band intensities in 4910 and 5310 cells with mean±SE of at least three individual experiments. B. Western blotting showing protein expression levels in mock, pSV and pM treatments. At 72 h post-transfection, cells were harvested and whole cell lysates were prepared using RIPA buffer. The representative blot of three different repetitions is shown. The blot was stripped and re-probed with anti-GAPDH antibody, which served as a loading control. The following bar diagram shows relative expression levels of MMP-2 protein with different treatments. C. Semiquantitative RT-PCR shows transcriptional levels of the MMP-2 gene and GAPDH was as a loading control. Band intensities were quantified using ImageJ 1.42 software (NIH Bethesda, USA) and the arbitrary units were plotted using mean±SE of at least three individual repetitions. D. Immunofluorescence study using blinded analysis showing the expression of MMP-2 in mock, pSV- and pM-treated 4910 and 5310 cells at 72 h post-transfection. After the treatments, cells were fixed in 4% paraformaldehyde, incubated with anti-MMP-2 antibody followed by Alexa Fluor® secondary antibodies, and observed under confocal microscopy. DAPI was used for nuclear counterstaining. Cells in randomly selected microscopic fields in three individual repetitions were represented where the fluorescence intensity was quantified using ImageJ and the arbitrary fluorescence units were plotted as mean±SE. The significant difference among different treatments in above experiments was represented by “**”, at *p*<0.01.

The article "Suppression of MMP-2 Attenuates TNF-α Induced NF-κB Activation and Leads to JNK Mediated Cell Death in Glioma" was retracted in 2025. Reasons: duplicated images; overlap with earlier publications; unreliable data; unreliable results or conclusions.

### MMP-2 downregulation leads to impeded proliferation and induces apoptosis *in vitro*

We next assessed the effect of pM on cell viability of 4910 and 5310 cells at different time intervals (24–96 h) using the MTT assay. We observed a time-dependent loss of cell viability significantly at 72 h of up to 61.4±4.2% in 4910 cells and 62.0±2.4% in 5310 cells (*p*<0.01). This effect was very prominent at 96 h with a significant loss of cell viability of up to 74.5±2.5% and 75.0±3.2% in 4910 and 5310 cells respectively, at *p*<0.01 (Fig. 2A). The FACS analysis to estimate the percent of apoptotic cells in the sub-G1 phase at the end of 72 h treatment revealed a remarkable cell death induced by pM. The percent of sub-G1 cells in pM-treated 4910 and 5310 cells was 32.8±1.2% and 33.9±1.8% respectively; whereas mock-treated cells only had 7.1±0.2% and 6.8±0.3% apoptotic cells and pSV-treated cells displayed a cell death rate of 6.7±0.3% and 7.4±0.15% (Fig. 2B). Analysis of DNA content indicated an increased proportion of cells in the G_2_-M phase after pM treatment. This could be due to cell cycle block in the G_2_-M phase or preferential apoptosis of these cells in late S and G_2_-M. Subsequently, to verify that this cell death was a result of apoptosis and to determine the mediators involved, we subjected whole cell lysates to Western blotting and determined cleavage of PARP, caspase-8 and caspase-3. These results clearly showed increased cleavage of PARP, caspase-8 and caspase-3 in the pM-treated cells when compared to the mock and pSV-treated controls, thereby implying that there is a significant hike in apoptotic cell death upon downregulation of MMP-2 in both of these cell lines (Fig. 2C). In addition, to confirm the apoptosis secondary to MMP-2 downregulation we determined extent of DNA fragmentation at 72 h post-transfection by TUNEL assay. In TUNEL assay, the apoptotic cells were significantly higher in pM-transfected cells when compared to mock and pSV treatments (Fig. 2D). The number of apoptotic cells were counted at 72 h post-transfection and percentage of TUNEL positive apoptotic cells was plotted in Fig. 2E, which shows up to 57.3±4.6% and 56.8±5.0% of the pM-transfected 4910 and 5310 cells were TUNEL-positive as compared to that of mock-treated (3.2±0.5% and 3.0±0.1%) and pSV-treated (3.3±0.36% and 2.8±0.5) cells, respectively. These results suggest that pM induced caspase-dependent apoptotic cell death.

The article "Suppression of MMP-2 Attenuates TNF-α Induced NF-κB Activation and Leads to JNK Mediated Cell Death in Glioma" was retracted in 2025. Reasons: duplicated images; overlap with earlier publications; unreliable data; unreliable results or conclusions.

**Figure 2:** MMP-2 RNA interference inhibited proliferation and induced apoptosis in human xenograft cell lines. A. 4910 and 5310 cells were treated with mock, pSV and pM for different time points (24 h, 48 h, 72 h and 96 h) and subjected to MTT cell viability assay. Data were represented as mean±SE of three independent experiments. The significant difference among different treatments was represented by “*”, at *p*≤0.05 and “**”, at *p*<0.01. B. Cell cycle distribution in 4910 and 5310 cells 72 h after mock, pSV and pM treatments. DNA content was analyzed by flow cytometry as described in Materials and Methods. The percentage of apoptotic population in cells was represented as G_0_ in histograms. Three individual experiments were conducted to confirm similar results. C. Whole cell lysates were prepared from mock, pSV- and pM-treated cells and subjected to Western blotting to check the cleavage of PARP, caspases-8 and caspases-3. Blots are representative of 3 independent experiments. D. Xenograft cell lines 4910 and 5310 were seeded in chamber slides and transfected with pSV and pM after 24 h for 72 hours at the end of which the cells were fixed in 4% paraformaldehyde and subjected to TUNEL assay. E. Percentage of apoptotic cells was plotted in corresponding bar diagrams with values representing mean±SE. and significant difference among treatments is represented by “**”, *p*<0.01.

### pM leads to decreased TNF-α expression and inhibits p65 phosphorylation and nuclear translocation via hindrance of IKKβ and phosphorylation of IκBα

The cytokine antibody array was performed using conditioned media to check the possible modulation of various cytokine levels in MMP-2siRNA treatments (data not shown). Among these we observed a striking inhibition in TNF-α levels in pM-treated conditioned medium when compared to conditioned medium in pSV treatment. Densitometric analysis showed up to ∼3 fold decreases in TNF-α levels upon MMP-2 depletion in both 4910 and 5310 cells. Western blotting using whole cell lysates confirmed the significant decrease of TNF-α expression in pM treated cells (Fig. 3A). With the prominent decrease in TNF-α expression, we next proceeded to determine the p65 phosphorylation levels in the cytosolic and nuclear fractions. There was drastic reduction in the phosphorylated p65 in the nuclear fractions of pM-treated cells when compared to either mock or pSV counterparts (Fig. 3B). The cytosolic phopsho-p65 levels also displayed remarkable decrease indicating that overall phosphorylation and subsequent nuclear translocation were inhibited in the pM-treated cells. To confirm this, localization of phospho-p65 was checked through confocal microscopy. In mock and pSV-treatments a higher phosphorylation levels of p65 were observed with the majority of staining resided in the nuclei indicating constitutive NF-κB activation in these cells. While the pM-treated cells showed significant loss of phospho-p65 with very little or no nuclear expression (Fig. 3C). Even though the inhibition in phosphorylation and nuclear translocation of p65 was evident at 24 h and 48 h post-transfection the inhibition was more prominent at the end of 72 h (data not shown). These results with evident inhibition of nuclear localization of p65 indicate that the MMP-2 depletion leads to a possible upstream change in NF-κB activating stimulus, which in turn, causes inhibition of its activation.

The article "Suppression of MMP-2 Attenuates TNF-α Induced NF-κB Activation and Leads to JNK Mediated Cell Death in Glioma" was retracted in 2025. Reasons: duplicated images; overlap with earlier publications; unreliable data; unreliable results or conclusions.

**Figure 3:** MMP-2siRNA induced inhibition of TNF-α mediated phosphorylation and nuclear translocation of p65 subunit of NF-κB in 4910 and 5310 xenograft cell lines. A. The 4910 and 5310 cells were transfected with either pSV or pM for 72 h as described in Materials and Methods. Conditioned medium (CM) was collected and subjected to cytokine array following manufacturer's instructions. The positive (Pos) and negative (Neg) controls show biotin-conjugated and non-biotinylated IgG respectively on the array. The tumor necrosis factor-alpha (TNF-α) levels in pSV (Scrambled Vector) control and pM (MMP-2siRNA) treatments were compared and relative intensity was estimated by densitometric analysis using ImageJ 1.42 (NIH). The arithmetic mean±SE values obtained from two independent repetitions were plotted in the bar diagram and significance was represented by “**”, at *p*<0.01. Whole cell lysates subjected to Western blotting to check the TNF-α expression levels. B. Cytoplasmic and nuclear extracts were subjected to Western blotting where HDAC-1 and GAPDH were used as internal controls for nuclear and cytosolic fractions, respectively. C. Immunocytochemistry showing the expression levels of phospho-p65 in mock, pSV and pM treated 4910 and 5310 cells. Cells were fixed in paraformaldehyde and incubated with anti-phospho-p65 antibody followed by Alexa Fluor® anti-rabbit secondary antibody, mounted and the expression levels and cellular localization of phospho-p65 were captured under a confocal microscope. The nucleus was counterstained with DAPI. D. The expression levels of IKKβ, IκBα, and pIκBα were determined in the whole cell lysates from mock, pSV- and pM-treated cells at 72 h post-transfection. Blots are representative of three independent experiments where GAPDH served as loading control.

The article "Suppression of MMP-2 Attenuates TNF-α Induced NF-κB Activation and Leads to JNK Mediated Cell Death in Glioma" was retracted in 2025. Reasons: duplicated images; overlap with earlier publications; unreliable data; unreliable results or conclusions.

The activation and nuclear translocation of NF-κB requires phosphorylation, ubiquitination and proteolytic degradation of IκBα by IKKβ. To determine the effect of pM on the phosphorylation of IκBα, we next determined the expression levels of IKKβ and total & phosphorylated IκBα levels using whole cell lysates. MMP-2 downregulation led to significant decrease in the IKKβ with simultaneous reduction in the expression levels of phosphorylated IκBα and elevation in total IκBα in both 4910 and 5310 cell lines (Fig. 3D). These results provide convincing evidence about the significant inhibitory effect of pM on the IKKβ-induced phosphorylation and degradation of IκBα and gives possible explanation for inhibited nuclear translocation of NF-κB through the IKKβ-IκBα pathway upon MMP-2 downregulation.

### Modulation of TRADD, TRAF2, FADD, Fas-L and Fas expression levels in pM treated cells

Further, to study the essential upstream events in the IKKβ-IκBα mediated NF-κB pathway involving intermediate adaptor proteins such as TRADD, RIP and TRAF-2, we next examined their expression levels and interaction using co-immunoprecipitation studies. We observed a significant decrease in the expression levels of TNFR1, TRADD, TRAF2 and RIP in pM-treated 4910 and 5310 cells. The FADD binds to activated Fas/Fas-L and facilitates recruitment of and activation of pro-casapse-8 leading to MAP kinase mediated cell death [20]. The Fas, Fas-L and FADD expression levels were remarkably elevated in pM-treated cells when compared to the controls suggesting a possible role of Fas signaling in pM-induced caspase-mediated cell death in these cells (Fig. 4A). The binding of TRADD and TRAF2 was decreased, as evident in the immunoprecipitation studies suggesting an inhibition in recruitment of TRAF2 to TRADD and giving a possible explanation for the inhibition of TRADD-TRAF2-mediated NF-κB activation in pM-treated cells (Fig. 4B). To further check the inhibitory role of MMP-2siRNA in TNF-α induced NF-κB activation, TNF-α was added to the culture medium to pM-transfected cells. The TNF-α treatment alone remarkably increased the p65 phosphorylation when compared to mock or pSV treated controls (Fig. 4C). On the other hand, the combination pM+TNF-α showed significant decrease in phopsho-p65 when compared to TNF-α treatment alone implying the role of TNF-α in MMP-2siRNA-inhibited p65 activation (Fig. 4D).

The article "Suppression of MMP-2 Attenuates TNF-α Induced NF-κB Activation and Leads to JNK Mediated Cell Death in Glioma" was retracted in 2025. Reasons: duplicated images; overlap with earlier publications; unreliable data; unreliable results or conclusions.

**Figure 4:** Inhibition of TNF-α mediated p65 phosphorylation by reduced interaction of TRADD-TRAF2. A. Whole cell lysates from mock, pSV- and pM-treated cells were subjected to Western blotting. Blots are representative of at least three independent experiments and blots were stripped and re-probed with GAPDH to check equal loading of samples. B. The immunoprecipitation experiments were performed by precipitating TRADD with anti-TRADD antibody or TRAF2 by using anti-TRAF2 antibody using μMACS™ protein G microbeads and MACS Separation Columns following manufacturer's instructions (Miltenyi Biotec, Germany). Immunoprecipitates were electrophoresed and probed with anti-TRADD or anti-TRAF2 antibodies to confirm the interaction. The non-specific IgG (Nsp-IgG) precipitates were loaded as negative control. C. The 4910 and 5310 cells were treated with mock, pSV, pM, and the combination treatments were performed by 10 ng/ml TNF-α treatment at the end of 60 h transfection to either mock or pM. Cells were further incubated for another 12 h and collected at the end of the experiment. Whole cell lysates were subjected Western blot analysis. The experiment was repeated thrice to verify results. D. The expression levels of phospho-p65 were quantified using ImageJ 1.42 (NIH) and plotted in the bar diagram with mean±SE values obtained from at least three individual repetitions. The significant difference among different treatments were indicated by “**”, at *p*<0.01.

### pM activates the MAP kinases p38 and JNK

To assess the expression levels of the MAP kinases after MMP-2 depletion, whole cell lysates were prepared at 24, 48 and 72 h post-transfection with pM and subjected to Western blotting. We observed dramatic increases in phosphorylated JNK and p38 levels after treatment with pM as compared to mock and pSV treatments in both 4910 and 5310 cells. We recorded a significant time-dependent prolonged activation of JNK of up to 72 h after transfection with up to 11-fold increase in phospho-JNK and up to 5 fold increase in phospho-p38; there was no change in expression of total JNK or p38 (Fig. 5A). The prolonged activation of JNK subsequently resulted in the elevation of phosphorylation of c-Jun. The simultaneous elevation in phospho-JNK and phospho-p38 MAPK and enhanced apoptotic response in transfected cells suggest a possible role of these molecules in pM-mediated cell death.

The article "Suppression of MMP-2 Attenuates TNF-α Induced NF-κB Activation and Leads to JNK Mediated Cell Death in Glioma" was retracted in 2025. Reasons: duplicated images; overlap with earlier publications; unreliable data; unreliable results or conclusions.

**Figure 5:** MMP-2 downregulation activated phosphorylation of MAP kinases and had a pro-apoptotic effect via activation of JNK. A. Whole cell lysates collected at different time points from mock, pSV- and pM-treated cells and were subjected to Western blotting. GAPDH was used as an internal control. Blots are representative of at least three independent experiments. B. The 4910 and 5310 cells were treated with mock, pSV and pM for 48 h and further treated with either SP600125 or SB203580 for another 24 h. At the end of 72 h cells were subjected to MTT cell viability assay. Data are presented as mean±SE and where significant difference among various treatment groups was represented by “*”, at *p*<0.05 and “**”, at *p*<0.01. C. Cells were collected at different time points (24 h, 48 h and 72 h) after pM transfection, and whole cell lysates were used to determine SAPK/JNK activity assay by quantitative immunoblotting using the non-radiolabeling method. Membranes were probed with phospho-c-jun (Ser 63). D. Individual treatments to 4910 and 5310 cells including mock, pSV and pM were carried out for 48 h followed by treatment with either SP600125 or SB203580 for another 24 h at the end of which cells were harvested. Whole cell lysates were subjected to Western blotting for cleavage of PARP, caspase-8 and caspase-3 and expression levels of phospho-JNK, JNK, phospho-p38 and p38. Representative blots from at least three independent experiments were shown.

### JNK inhibitor, but not p38 inhibitor, reverses pM-induced cell death

Sequentially, to investigate the possible involvement of enhanced phospho-JNK and phospho-p38 in pM-induced cell death, we performed combination treatments of mock, pSV and pM with JNK inhibitor II (SP600125) or p38 MAPK inhibitor (SB203580) as described previously. Cell viability in individual experiments was determined to assess the reversal of pM-induced cell death by these inhibitors. In the combination treatment of pM+SB203580 there was no significant reversal of loss of cell viability with SB203580 treatment, which indicates that there was no obvious role of enhanced p38 MAPK phosphorylation in pM-induced apoptosis (Fig. 5B). However, JNK phosphorylation inhibition by SP600125 supplementation to pM treatment remarkably increased cell viability by blocking pM-induced cell death in both 4910 (from pM; 36.6±2.8 to pM+SP600125; 61.5±1.5%) and 5310 (from pM; 35.5±2.0 to pM+SP600125; 62.6±3.3%) cells (*p*<0.05). While, the supplementation of either SB203580 or SP600125 on mock and pSV treatments showed similar response on cell viability as that of mock and pSV suggesting that the addition SP203580 has no or little effect on cell death. These results clearly indicate an apparent role of JNK activation in pM-mediated cell death. With the elevated and prolonged phosphorylation of JNK, we next proceeded to determine JNK activity using c-Jun fusion protein coated beads after pM treatments. We noted a gradual, time-dependent significant increase in JNK activity as observed by enhanced c-Jun phosphorylation, which resulted in increasing phosphorylation of c-Jun in both cell lines upon MMP-2 depletion from 24 to 72 h (Fig. 5C). The mock and pSV treatments did not show any time dependent elevation of JNK activity (data not shown). We next assessed the affect of enhanced p38 and JNK phosphorylation on pM induced cell death through combination experiments mock, pSV and pM in conjunction with SP600125 and SB203580 by subjecting whole cell lysates to Western blot analyses for identifying the cleavage of apoptotic molecules. In corroboration with the cell viability assays, Western blotting clearly indicated that the enhanced cleavage of PARP, caspase-8, and caspase-3 by treatment with pM alone was compromised in these cells when treated with SP600125, suggesting a significant reversal of cleavage of apoptotic molecules in combination of pM+SP600125. However, treatment with SP600125 alone led to decreased caspase cleavage as compared to mock treatments, implying blocking of prolonged JNK phosphorylation in pM-treated cells protects these cells from JNK-induced cell death (Fig. 5D). On the other hand, treatment with p38 inhibitor SB203580 along with pM did not significantly reversed the pM-induced cell death which is evident from the cleavage of apoptotic molecules in combination treatment comparable to the pM treatment alone. The treatments with either SP600125 or SB203580 alone did not show any effect on phospho-p38 and phospho-JNK respectively (Fig. 5D).

The article "Suppression of MMP-2 Attenuates TNF-α Induced NF-κB Activation and Leads to JNK Mediated Cell Death in Glioma" was retracted in 2025. Reasons: duplicated images; overlap with earlier publications; unreliable data; unreliable results or conclusions.

### Supplementation of rhMMP-2 rescued 4910 and 5310 cells from pro-apoptotic effect of pM and reversed the inhibited NF-κB DNA binding activity

To further confirm that the observed apoptosis in our experiments was caused by specific downregulation of MMP-2 and not due to any off-target consequences, we supplemented cells with recombinant human MMP-2 (rhMMP-2). We observed a significant dose-dependent elevation in MMP-2 expression in both 4910 and 5310 cells when rhMMP-2 was added into the medium. We chose an optimized concentration of 25 ng/ml rhMMP-2 for combination treatments (data not shown). The reversal of MMP-2 downregulation and subsequent apoptosis upon the addition of rhMMP-2 was confirmed by Western blotting. MMP-2 expression hampered by pM treatment was overturned upon supplementation of rhMMP-2 in both 4910 and 5310 cells. As noted earlier, pM induced cleavage of PARP, caspase-8 and caspase-3; this cleavage was reduced in rhMMP-2-treated cells as compared to either mock or pSV-treated cells. The combination treatment of pM+rhMMP-2 reversed the PARP, caspase-8 and -3 confirming the pro-apoptotic function of pM treatment in both cell lines (Fig. 6A). The relative intensities of cleaved caspase-8 and caspase-3 were quantified and plotted in the bar diagram which clearly showed the significant reversal of elevated caspase cleavage in the combination treatment (Fig. 6B). Western blotting showed elevated expression of TNF-α and TRADD in the rhMMP-2 treated cells and the inhibition of these molecules by pM treatment alone was significantly reversed in the combination treatment. The IKKβ and pIκBα were subsequently elevated in rhMMP-2 treatment and a significant reversal in the combination of pM+rhMMP-2 (Fig. 6C). Similarly, the treatment of pM with augmentation of rhMMP-2 restored the nuclear expression levels of phospho-p65 in pM-treated 4910 and 5310 cells, whereas rhMMP-2 alone significantly enhanced the nuclear levels of phospho-p65 (Fig. 6D). In addition, to determine the effect of these treatments on NF-κB DNA binding activity nuclear extracts from individual treatments of mock, pSV, pM, rhMMP-2 and pM+rhMMP-2 were used to perform EMSA. The results in Figure 6E clearly show that pM significantly reduced DNA-binding activity when compared to mock and pSV-treated 4910 and 5310 cell lines while rhMMP-2 treatment alone enhanced DNA binding activity. Moreover, supplementation rhMMP-2 to pM-treated cells restored the pM-inhibited NF-κB DNA binding activity (Fig. 6E). We carried out the TUNEL assay to further check the possible reversal of pM-induced apoptotic cell death by either SP600125 or rhMMP-2. These clearly indicated a significant reversal of pM-induced cell death by the treatment with either SP600125 or rhMMP-2 in both cell lines (Fig. S1). The percentage of apoptotic cells was plotted which showed a significant reversal pM-induced cell death by SP600125 and rhMMP-2 while the treatment with SP600125 and rhMMP-2 showed decreased cell death when compared to either mock or pSV controls (*p*<0.05) (Fig. 7A).

**Figure 6:** Effect of rhMMP-2 treatment on pM-inhibited NF-κB activity. A. The 4910 and 5310 cells were transfected with mock, pSV and pM for 48 h and treated with 25 ng/ml rhMMP-2 for another 24 h. Whole cell lysates from mock, pSV, pM, rhMMP-2, pM+rhMMP-2 treatments were prepared at the end of 72 h experiment and subjected to Western blotting to check the expression levels of MMP-2, and cleavage of PARP, caspase-8 and caspase-3. B. The relative intensity of cleaved caspase-8 and caspase-3 were quantified using ImageJ (NIH) software and plotted in the bar diagram using mean±SE and significant difference was represented by “**”, at *p*<0.01. C. The expression levels of TNF-α, TRADD, IKKβ and, p-IκBα were checked for the possible reversal and upregulation of IKKβ-pIκBα mediated NF-κB pathway. D. The nuclear fractions were checked for phospho-p65 expression levels in pM+rhMMP-2 combination treatment where HDAC-1 served as nuclear and loading control. E. Electrophoretic mobility shift assay showing the DNA binding activity of p65. Nuclear extracts at the end of 72 h were prepared from the mock, pSV, pM, rhMMP-2, pM+rhMMP-2 treatments as described above in 4910 and 5310 cells and subjected to EMSA where rhMMP-2+p65α antibody was loaded to check the shift and cold probe was loaded as negative control.

The article "Suppression of MMP-2 Attenuates TNF-α Induced NF-κB Activation and Leads to JNK Mediated Cell Death in Glioma" was retracted in 2025. Reasons: duplicated images; overlap with earlier publications; unreliable data; unreliable results or conclusions.

**Figure 7:** A. Effect of JNK inhibitor (SP600125) and recombinant human MMP-2 (rhMMP-2) treatment on pro-apoptotic effect of MMP-2 downregulation. The number of TUNEL positive cells were scored in randomly selected microscopic fields at the end of various treatments as described in Materials and Methods. The percentage of apoptotic cells in each treatment was plotted in bar diagrams with mean±SE and significant difference among various treatment groups was represented by “*”, at *p*<0.05 and “**”, at *p*<0.01 in three individual repetitions. B. Effect of rhMMP-2 treatment on pM induced FADD, Fas, Fas-L and pJNK expression. The whole cell lysates from different treatments were subjected to Western blotting. C. Role of Fas in pM induced JNK activation. The Fas/Fas-L function was blocked by using neutralizing antibody against Fas in the individual treatments. At the end of 60 h transfection, anti-Fas ab (250 ng/ml) was added and cells were further incubated for another 12 h at the end of which whole cell lysates were prepared and subjected to Western blotting to determine the effect of Fas/Fas-L functional blocking on JNK phosphorylation. The blots are representative of three individual experiments.

### Role of Fas activation in pM-induced JNK activation

Our previous studies with specific MMP-2 downregulation showed the elevation of TIMP-3, which in turn cleaves Fas-L and activated Fas/Fas-L apoptotic signaling in lung adenocarcinoma cells [31]. In corroboration with this report, we observed remarkably enhanced TIMP-3 levels in pM treatment and the enhanced TIMP-3 levels were reversed in the combination of pM+rhMMP-2 (Fig. S2). To assess the possible role of Fas/Fas-L activation in MMP-2 inhibition induced JNK mediated cell death in 4910 and 5310 cell lines, rhMMP-2 was supplemented and whole cell lysates were analyzed for the possible reversal of pM-induced Fas mediated JNK activation. The expression of FADD, Fas and Fas-L and phosphorylation of JNK was reduced in the rhMMP-2 alone when compared to either mock or pSV, which implies a correlation with the increased cell viability in rhMMP-2 in both 4910 and 5310 cell lines. On the other hand, the rhMMP-2 supplementation to pM-treated cells counteracted on the pM-induced FADD, Fas, Fas-L and phospho-JNK expression levels with no substantial change in the total JNK (Fig. 7B). Subsequently, to confirm the role of Fas signaling in the activation of JNK, we performed a Fas functional blocking experiment with anti-Fas ab. When the treatment with anti-Fas antibody was compared to either mock or pSV treatment, there was an evident decrease in the phosphorylation of JNK with the specific blocking of Fas activation which showed the Fas-mediated JNK activation in these glioma xenograft cells (Fig. 7C). In contrast, when Fas activation was blocked in the pM-treated cells there was a significant reversal of the elevated JNK phosphorylation, suggesting a role of Fas activation in JNK mediated cell death in MMP-2 downregulated 4910 and 5310 cells.

The article "Suppression of MMP-2 Attenuates TNF-α Induced NF-κB Activation and Leads to JNK Mediated Cell Death in Glioma" was retracted in 2025. Reasons: duplicated images; overlap with earlier publications; unreliable data; unreliable results or conclusions.

### MMP-2siRNA treatment regressed tumor growth *in vivo*, induces apoptosis with decreased phospho-p65 and elevated expression of phospho-JNK levels

We next proceeded to determine the effect of pM on tumor growth *in vivo*. The brain tumor sections were prepared as described above and the mock, pSV and pM samples were evaluated histologically for tumor formation and expression levels of various proteins. Compared to mock and pSV-treated tumors, tumor development was remarkably regressed in pM-treated mice (Fig. 8A). We observed a significant reduction in the relative tumor size at *p*<0.01 (Fig. 8B). We next evaluated the tumors for the expression of MMP-2, phospho-p65 and phosho-JNK. In mock and pSV-treated tumors, we observed high MMP-2 expression whereas we observed very less MMP-2 expression in pM-treated tumors (Fig. 8C). Further, immunostaining confirmed the high phosphorylation levels of p65 in mock and pSV-treated tumor sections which directly indicates the constitutive NF-κB activity in these tumor cells, while pM treatment resulted in significant inhibition of phospho-p65 expression levels (Fig. 8D). Moreover, a significantly elevated expression of phospho-JNK was observed in pM-treated tumors when compared to mock and pSV-treated tumors (Fig. 8E). The results of the TUNEL assay indicate that pM treatment resulted in induction of apoptosis as evident from the elevated number of TUNEL-positive cells whereas very few TUNEL or no TUNEL-positive apoptotic cells were observed in mock and pSV-treated tumors (*p*<0.01) (Fig. 8F,G). These *in vivo* results corroborate our *in vitro* results.

The article "Suppression of MMP-2 Attenuates TNF-α Induced NF-κB Activation and Leads to JNK Mediated Cell Death in Glioma" was retracted in 2025. Reasons: duplicated images; overlap with earlier publications; unreliable data; unreliable results or conclusions.

**Figure 8:** Tumorigenicity *in vivo* in nude mice (nu/nu) brains induced by intracranial injection of 4910 and 5310 cells. The pSV and pM plasmids were injected into the tumors as described in Materials and Methods while the 1×PBS injection served as the mock control treatment. At the end of the experiment the brains were removed and fixed in 10% phosphate-buffered formaldehyde and the fixed tissue samples were subsequently embedded in paraffin blocks. A. Hematoxylin and Eosin staining of brain sections displaying the neoplastic growth of tumors after injections of 4910 and 5310 cells (10× and 60×). B. The tumor area from every fifth H&E stained tumor section was calculated with the aid of microscope attached computer screen and Image Pro Discovery Program software (Media Cybernatics, Inc., Sliver spring, MD). The total tumor volume is calculated as summed area of tumor on all sections multiplied by width of the sections. The relative brain tumor size was estimated from mock-pSV and pM treated animals and plotted as mean±SE obtained from a group of 10 animals. The significant difference among different treatment groups was represented by “**”, at *p*<0.01. C. Immunohistochemical analyses through DAB staining were performed to detect the expression of MMP-2 in paraformaldehyde embedded tumor sections. Hematoxylin was used for nuclear counter staining and rabbit IgG was used as a negative control. D, E. Immunohistochemical studies showing the expression of phospho-p65 and phospho-JNK in mock, pSV, pM treated tumor sections. Hematoxylin was used for nuclear counter-staining and rabbit IgG was used a negative control. F. Examination of *in situ* cell death by TUNEL assay of brain tumor cells after treatments. Rabbit IgG was used as a negative control. G. Total number of apoptotic cells was counted in randomly selected microscopic fields and plotted in bar diagram with mean±SE and significant difference among treatment groups was represented by “**”, at *p*<0.01.

## Discussion

Extensive endothelial proliferations, robust growth and further dissemination of tumor cells are the consequences of extracellular matrix and basement membrane disruption, which is in part mediated by the action of MMPs [6]. In the present study, we demonstrate that the transcriptional inactivation of MMP-2 induced apoptosis in human xenograft cell lines *in vitro* and *in vivo* through suppression of the NF-κB and activation of JNK.

The article "Suppression of MMP-2 Attenuates TNF-α Induced NF-κB Activation and Leads to JNK Mediated Cell Death in Glioma" was retracted in 2025. Reasons: duplicated images; overlap with earlier publications; unreliable data; unreliable results or conclusions.

TNF-α mediates its downstream effects by transducing signals to different effectors, including IKK, JNK and caspases [10]. It is noteworthy that IKK activation inhibits caspase-mediated apoptosis through the transcription factor NF-κB, whose target genes includes caspase inhibitors. Several lines of evidence suggest the existence of negative cross-talk between the NF-κB and the JNK pathways. Previous studies have demonstrated that, in mouse embryonic fibroblasts that are deficient of the catalytic subunit IKKβ or p65, the IKK/NF-κB pathway negatively regulates TNF-α-mediated JNK activation partly through the upregulation of NF-κB-induced XIAP and gadd45beta/myd118 [10]. Our studies with TNF-α treatment showed p65 downregulation in MMP-2siRNA treatments indicating a possible role of MMP-2 in the regulation TNF-α induced NF-κB activation. RIP is part of the TNFR1 complex and consists of three domains: death domain, S/T kinase homology domain, and poorly conserved intermediate domain where the death domain of RIP facilitates its interaction with the death domain of CD95 (Fas/APO-1), which is responsible for apoptotic induction while the intermediate domain is essential for activation of NF-κB [10], [23], [33]. In addition, previous researchers have demonstrated that the death domain of RIP is sufficient to induce apoptosis, and RIP^−/−^ cells were unresponsive to TNF-α stimulated NF-κB activation. RIP is cleaved into RIPn (containing the entire kinase domain) and RIPc fragments by the action of caspase-8, which results in inhibition of TNF-α-induced NF-κB activation and induces apoptosis probably through enhancing the interaction of TRADD and FADD [21]–[23]. Our current study demonstrating RIP downregulation in MMP-2 depletion suggests a possible role of MMP-2 in the RIP mediated NF-κB signaling activation.

We observed a significant decrease in the expression levels of TNF-α, TNFR1, TRADD and TRAF2 and immunoprecipitation experiments revealed inhibited interaction of TRADD-TRAF2 and along with increased FADD expression levels in pM-treated 4910 and 5310 glioma xenograft cells. The decreased TRADD-TRAF2 interaction might lead to the inhibition of downstream IKKβ mediated NF-κB activation. These results are in corroboration with the previous report on MMP-2 depletion induced decrease in TRADD in 4910 cells [32]. FADD was originally identified as an important molecule for Fas-mediated apoptosis and is an important component in DISC. DISC, which is at least composed of FADD, caspase 8 and Fas, activates pro-caspase-8, which subsequently activates effector caspases (e.g., caspase-3) whose activation results in the induction of apoptosis [34]. Recent reports suggest that FADD induced apoptosis by modulating different effector molecules, especially by activating the JNK signaling pathway. Overexpression of constitutively active JNK or its upstream kinases led to the induction of apoptosis via caspase activation, whereas overexpression of dominant negative forms resulted in the inhibition of apoptosis. Further, JNK is also essential for activating Fas-mediated death signaling and responsible for sensitization to apoptosis induced by various drugs [35]–[37]. FADD phosphorylation, which is a major event in the chemosensitization to various DNA damaging agents, at the G_2_/M check point leads to cell cycle arrest [38]. This phosphorylation is dependent on JNK signaling, and in turn, FADD promotes JNK signaling activation [39]. The negative regulation of TNF-α on Fas-induced apoptosis in tumor cells has been previously reported in tumor cells [40], [41]. Our previous studies with specific suppression of MMP-2 in lung cancer cells demonstrated the upregulation of TIMP-3 mediated Fas/Fas-L apoptotic pathway. In corroboration with these studies, our current study using MMP-2siRNA shows that the inhibition of MMP-2 resulted in the elevation of TIMP-3, FADD, Fas, Fas-L and cleavage of caspase-8, -3 and PARP with simultaneous JNK activation. The specific functional blocking of Fas activation led to suppressed pM-induced JNK activation confirming the role of Fas/Fas-L in the JNK mediated cell death in these glioma xenograft cells. In our study, both *in vitro* and *in vivo* animal experiments showed JNK activation with pM treatments and which subsequently led to apoptosis as determined by TUNEL assay. Reversal experiments with SP600125 for JNK inhibition corroborate previous reports on JNK-induced cell death through the activation of caspases. In contrast to JNK, treatments with SB203580 to inhibit p38 MAPK; our results show that p38 activation did not play a role in pM-induced cell death. On the other hand, the addition of rhMMP-2 led to enhanced DNA-binding activity of NF-κB by elevating TRADD expression levels suggesting a role of MMP-2 in the regulation of NF-κB signaling. In consistency with our *in vitro* findings, pM treatment regressed intracranial tumor development and activated JNK and inhibited NF-κB nuclear expression levels in *in vivo* experiments. Here, our results suggest a model where MMP-2 depletion using MMP-2siRNA modulates TRADD, TRAF2 interactions, which in turn, leads to NF-κB inhibition and Fas/Fas-L induced JNK mediated apoptosis. The present study provides auxillary insights into the molecular mechanisms underlying siRNA-mediated MMP-2 downregulation and suggests the potential value of MMP-2 as a therapeutic target in the treatment of glioma.

The article "Suppression of MMP-2 Attenuates TNF-α Induced NF-κB Activation and Leads to JNK Mediated Cell Death in Glioma" was retracted in 2025. Reasons: duplicated images; overlap with earlier publications; unreliable data; unreliable results or conclusions.

## Materials and Methods

### Ethics Statement

The Institutional Animal Care and Use Committee of the University of Illinois College of Medicine at Peoria, Peoria, IL, USA, approved all surgical interventions and post-operative animal care. The consent was written and approved. The animal protocol number is 858, dated May 27, 2009, and renewed on April 27, 2010.

### Chemicals and antibodies

We used antibodies specific for MMP-2, TNF-α, TNFR1, TRADD, RIP, TRAF-2, FADD, p65, and phospho-p65 (Ser536), phospho-JNK (Ser63), JNK1, phospho-p38 MAPK (Tyr182), p38 MAPK, phospho-c-Jun (Ser73), c-Jun, GAPDH (Santa Cruz Biotechnology, Santa Cruz, CA), IKKβ, IκBα, phospho-IκBα (Ser32), poly (ADP-Ribose) polymerase, caspases-3 and caspases-8 (Cell Signal Technology, Boston, MA), HRP/Alexa Fluor® conjugated secondary antibodies (Santa Cruz Biotechnology, Santa Cruz, CA). We also purchased p38 MAPK inhibitor (SB203580) and JNK inhibitor II (SP600125) (Calbiochem, La Jolla, CA), anti-Fas (human, neutralizing clone ZB4) antibody (Millipore, Temecula, CA) and human recombinant-MMP-2 protein (EMD Biosciences, San Diego, CA) and used in this study.

### Cell culture, Plasmid vector and transient transfection studies

The 4910 and 5310 human xenograft cell lines (kindly provided by Dr. David James, University of California at San Francisco), were generated and maintained in mice and are highly invasive in the mouse brain [42]. Cells were cultured in RPMI 1640 (Mediatech Inc., Herndon, VA) supplemented with 10% fetal bovine serum (Invitrogen Corporation, Carlsbad, CA), 50 units/ml penicillin, and 50 µg/ml streptomycin (Life Technologies, Inc., Frederick, MD) in a humidified 5% CO_2_ chamber maintained at 37°C. The siRNA sequence specific for MMP-2: AACGGACAAAGAGTTGGCAGTATCGATACTGCCAACTCTTTGTCCGTT was designed and cloned in CMV promoter driven mammalian transfection vector, pcDNA3.1(+) (pM) at *Nhe*I site where as pcDNA3.1 (+) vector containing a specific scrambled sequence for MMP-2 siRNA (pSV): GCACGGAGGTTGCAAAGAATAATCGATTATTCTTTGCAACCTCCGTGC, served as negative control along with mock (1×PBS) treatment. Transient transfection studies were performed using FuGene HD transfection reagent as per the manufacturer's instructions (Roche Applied Science, Indianapolis, IN) as describes previously [30]. Briefly, up to 70% confluent cells were serum-starved for 6 h after which they were transfected with mock, pSV and pM, and were harvested at 24 h, 48 h, 72 h and 96 h post-transfection and used for further molecular analyses. For combination treatments, JNK inhibitor (SP600125; 10 µM), p38 inhibitor (SB203580; 10 µM) or recombinant human MMP-2 (rhMMP-2; 25 ng/ml) protein were supplemented in the medium to cells at 48 h pM post-transfection and the cells were incubated for another 24 h. For the TNF-α and anti-Fas functional blocking treatment, at 60 h post-transfection either TNF-α (10 ng/ml) or anti-Fas (250 ng/ml) were added and incubated for another 12 h at the end of which cells were collected.

The article "Suppression of MMP-2 Attenuates TNF-α Induced NF-κB Activation and Leads to JNK Mediated Cell Death in Glioma" was retracted in 2025. Reasons: duplicated images; overlap with earlier publications; unreliable data; unreliable results or conclusions.

### Gelatin zymography

The gelatinolytic activity of MMP-2 using conditioned media was measured as described previously [30]. In short, 60 h after transfection of mock, pSV and pM, 3 mL of serum-free medium were added, and cells were incubated for another 12 h and the conditioned media were resolved over 0.1% gelatin-SDS-polyacrylamide gels. Gels were washed in 2.5% Triton X-100 to remove SDS, followed by an overnight incubation at 37°C in Tris-CaCl_2_ buffer (pH-7.6) and stained with Coomassie brilliant blue. The gelatinolytic activity of the protein was visualized through negative staining as clear sectors of lyses against a dark blue backdrop.

### RNA isolation and Reverse transcriptase polymerase chain reaction (RT-PCR)

Total RNA from mock, pSV- and pM-treated cells was extracted at 72 h post-transfection using TRIzol reagent (Invitrogen) as per the manufacturer's instructions. The ImProm-II Reverse Transcription (Promega Corporation, Madison, WI) along with 2 µg of total RNA and poly-dT primers were used for synthesis of cDNA. To determine the RNA transcript levels from cDNA, PCR was carried out with 1 µL of cDNA using the following primers: for MMP-2 sense 5′-GTGCTGAAGGACACACTAAAGA-3′ and antisense 5′-CCTACAACTTTGAGAAGGATGGCAA-3′, and for GAPDH sense 5′- GGAGTCAACGGATTTGGTCGTAT -3′ and antisense 5′- GTCTTCACCACCATGGAGAAGGCT -3′. The PCR conditions were as follows: initial denaturation at 95°C for 3 min, followed by 30 cycles at 95°C for 1 min, 58°C for 30 sec, 72°C for 45 sec, followed by a final extension at 72°C for 10 min. Amplified PCR products were visualized in ethidium bromide agarose gels under ultraviolet light.

### Preparation of cytoplasmic and nuclear extract

Cells were treated with mock, pSV, pM, SP600125, pM+SP600125, rhMMP-2, or pM+rhMMP-2 for 72 h as described above, collected and washed twice with ice-cold PBS. The nuclear and cytoplasmic proteins were prepared using the Biovision Nuclear/Cytosol Fractionation Kit (Mountain View, CA) as per manufacturer's instructions and used in further analyses [43].

### Western blotting, immunoprecipitation and cytokine antibody array

Cells were harvested at the end of different treatments and lysed in radioimmunoprecipitation assay (RIPA) buffer containing protease inhibitors as described previously [31]. For immunoprecipitation, quantified whole cell lysates were precipitated with anti-TRADD antibody using μMACS™ protein G microbeads and MACS Separation Columns following manufacturer's instructions (Miltenyi Biotec, Germany). Equal amounts of protein fractions or immunoprecipitates of lysates with indicated antibodies were resolved over SDS-PAGE and transferred on to PVDF membrane. Blots were incubated in respective primary antibodies followed by incubation in HRP-conjugated secondary antibodies and subsequently exposed to autoradiography. The Human Cytokine Array 3 kit was used to verify relative levels of cytokines released from 4910 and 5310 cells after pSV and pM treatments using conditioned media following manufacturer's instructions (Ray Biotech®, Norcross, GA) as described previously [44]. Each cytokine was present in duplicate on the array in the form of dots and the array was repeated thrice to confirm similar results. The average signal intensities of both dots for expression analysis of each cytokine were compared where biotin-conjugated IgG was used for positive signal. Differential changes in cytokine production were calculated by densitometric analysis using ImageJ 1.42 (NIH) software.

The article "Suppression of MMP-2 Attenuates TNF-α Induced NF-κB Activation and Leads to JNK Mediated Cell Death in Glioma" was retracted in 2025. Reasons: duplicated images; overlap with earlier publications; unreliable data; unreliable results or conclusions.

### Electrophoretic mobility shift assay

Nuclear extracts from mock, pSV, pM, rhMMP-2 and pM+rhMMP-2 treated cells were analyzed using the electrophoretic gel shift assay. The anti-p65 (p65α) antibody was added to check the specificity and cold probe served as a negative control. The complexes of protein–biotin labeled p65 binding DNA were resolved on a 5% non-denaturing gel, subsequently transferred onto N^+^ membrane, and subjected to autoradiography as per the manufacturer's instructions (Panomics EMSA Kit, Panomic, Inc. Fremont, CA).

### JNK activity assay

A non-radiolabeling quantitative immunoblotting SAPK/JNK Kinase Assay Kit (Cell Signal Technology, Boston, MA) was used to perform the JNK activity assay. Cells were treated with mock, pSV or pM and whole cell lysates were prepared and immobilized, and c-Jun fusion protein bead slurry was added as described in the manufacturer's protocol. The samples were incubated overnight at 4°C and subsequently centrifuged and the pellet was incubated with 500 µL kinase buffer and 200 µM ATP for 30 min at RT. The samples were resolved on SDS-PAGE and transferred onto the PVDF membrane and Western blotting was carried out to detect phosphorylated c-Jun.

### MTT assay

The 4910 and 5310 cells (1×10^3^/well) were plated in a 96-well plate and incubated overnight. Treatments of mock, pSV, pM in combination either SP600125 or SB203580 were carried out for 72 h as described above. Cell viability was determined by MTT assay as described earlier [41]. Absorbance was read at 590 nm using a 96-well microplate reader.

The article "Suppression of MMP-2 Attenuates TNF-α Induced NF-κB Activation and Leads to JNK Mediated Cell Death in Glioma" was retracted in 2025. Reasons: duplicated images; overlap with earlier publications; unreliable data; unreliable results or conclusions.

### Flow cytometry

Cells were transfected with mock, pSV or pM as described above and were harvested after 72 h and fixed in 70% ethanol for 1 h at 4°C. Subsequently, the cells were stained with propidium iodide (BioSure, Grass Valley, CA) for 30 min in the dark and FACS analysis was performed using a Becton-Dickinson FACS Calibur flow cytometer (BD Biosciences, Heidelberg, Germany). Results were analyzed with Cell Quest software (BD Biosciences, Heidelberg, Germany).

### In situ terminal deoxynucleotidyl transferase dUTP nick end labeling (TUNEL) assay

The apoptotic population of mock, pSV- and pM-treated cells or paraformaldehyde fixed and paraffin embedded mice brain tumor sections from 4910/5310 xenograft cells was detected using a TUNEL apoptosis detection kit (Roche Diagnostics, Indianapolis, IN) following manufacturer's protocol. Samples were incubated in TUNEL reaction mixture containing TdT and fluorescein-dUTP at 37°C for 1 h where TdT catalyses the binding of fluorescein-dUTP to free 3′OH ends in the nicked DNA. The cells were visualized for the incorporated fluorescein under confocal microscope.

### Immunocytochemical and immunohistochemical analyses

Immunocytochemical and immunohistochemical analyses were performed as described earlier [41]. The transfected 4910 and 5310 cells in chamber slides were fixed in paraformaldehyde followed by permeabilization in 0.1% Triton-X100. Non-specific binding was blocked in 1% BSA in PBS, followed by incubation with anti-MMP-2 and anti-p65 antibodies for 2 h at room temperature. The cells were washed and incubated with Alexa Fluor®-conjugated secondary antibodies, subsequently mounted. For nuclear counterstaining, 4′-6-diamidino-2-phenylindole (DAPI) was used. For immunohistochemical analysis, tissue sections (4–5 µm) were de-paraffinized in xylene, rehydrated in graded ethanol solutions, permeabilized in 0.1% Triton X-100, and incubated overnight at 4°C with anti-MMP-2, anti-phospho-p65 and anti-phospho-JNK antibodies. Slides were washed twice in PBS and incubated in either Alexa Fluor®- or HRP-conjugated secondary antibodies for 1 h at room temperature followed by counterstaining with DAPI. For DAB staining, the HRP-conjugated secondary antibodies incubated sections were washed and further incubated with DAB (3,3′-Diaminobenzidine) solution for 5–10 min while Hematoxylin was used for nuclear counterstaining, mounted and photographed under a microscope.

### In-vivo experiments

The 4910 and 5310 cells (2×10^6^ cells/100 µL) were injected sterotactically into athymic, female, 4–6-week old ***nu/nu*** mice as described previously [30]. After 10 days, the animals were divided into three sets (n = 10) and ALZET osmotic pumps (model 2004, ALZET® Osmotic Pumps, Cupertino, CA) were implanted for plasmid delivery (dose: 6 mg/kg body weight). Animals losing >20% of the body weight or having problems in feeding and grooming were euthanized. Animals were observed up to 60 days at the end of which brains were excised and fixed in 10% buffered formalin, and embedded in paraffin. To visualize tumor cells and to examine tumor development, the brain sections were stained with H&E. The tumor area from every fifth H&E stained tumor section was calculated with the aid of microscope attached computer screen and Image Pro Discovery Program software (Media Cybernatics, Inc., Sliver spring, MD). The total tumor volume is calculated as summed tumor area on all sections multiplied by width of the sections. The relative brain tumor size was estimated from mock-pSV and pM treated animals and plotted as mean±SE obtained from a group of 10 animals.

The article "Suppression of MMP-2 Attenuates TNF-α Induced NF-κB Activation and Leads to JNK Mediated Cell Death in Glioma" was retracted in 2025. Reasons: duplicated images; overlap with earlier publications; unreliable data; unreliable results or conclusions.

### Statistical analysis

Data obtained from different treatment groups were analyzed using one-way ANOVA by Neumann-Keuls method of Sigmastat 3.1. The relative expression or fluorescence intensities were quantified using ImageJ 1.42 software (NIH, U.S.A.). Data were represented in the form of mean±SE, which was obtained from at least three individual repetitions and the significant difference among different treatment groups was denoted by “*”, at *p<*0.05 and “**”, at *p<*0.01.

## Supporting Information

Figure S1 **Effect of rhMMP-2 and JNK inhibition by SP600125 treatment on pM-induced apoptosis.** Representative images show apoptotic cell death by TUNEL assay in three individual repetitions at the end of 72 h in 4910 and 5310 cells.
(TIF)

Figure S2 **Western blotting showing the expression levels of TIMP-3 in mock, pSV, pM, rhMMP-2, pM+rhMMP-2 treatments in 4910 and 5310 cells.**
(TIF)
